# Effects of Tai Chi Softball Exercises on Physical Fitness Level and Cardiovascular Health-Related Factors among Older Females

**DOI:** 10.1155/2021/7671596

**Published:** 2021-07-02

**Authors:** XiaoDong Cheng, Yongzhao Fan, Ling Ge, Desen Zang, Jianxi Li, Jian Li, Hao Wu

**Affiliations:** ^1^Capital University of Physical Education and Sports, Beijing 100191, China; ^2^Comprehensive Key Laboratory of Sports Ability Evaluation and Research of the General Administration of Sport of China, Beijing Key Laboratory of Sports Function Assessment and Technical Analysis, Beijing 100191, China; ^3^Hefei No. 10 Middle School, Hefei 230001, Anhui, China; ^4^Winter Games Management Center, Xi'an 710061, Shaanxi, China

## Abstract

Tai Chi softball was voted as one of the most popular health-promoting exercises and can also develop manipulative skill and hand-eye coordination. The purpose of this study was to explore changes in the physical fitness level and cardiovascular health-related factors after the 16-week Tai Chi softball (TCSB) training program among older females. One hundred healthy older females were assessed at the baseline before TCSB training, and then, they conducted intervention experiments. Through the 16-week TCSB intervention training, a control group and a physical exercise group showed significant differences. The physical exercise group significantly reduced body mass index, systolic blood pressure, and diastolic blood pressure from all the results studied. It also reduces total cholesterol, triglycerides, low-density lipoprotein cholesterol (^*∗*^*p* < 0.05), and waist-to-hip ratio (^*∗∗*^*p* < 0.01), whereas handgrip, sit and reach, single leg stance, vital capacity (^*∗*^*p* < 0.05), and high-density lipoprotein cholesterol (^*∗∗*^*p* < 0.01) were significantly increased. TCSB training may improve physical fitness ability and decrease the risk of cardiovascular disease among older females.

## 1. Introduction

The global proportion of the elderly is constantly increasing. From 2015 to 2020, the proportion of people over 60 has nearly doubled. There is a general lack of physical exercise in this age group [1]. For example, older females (OF) with less activity spent more time sitting (10–15 hours/day) than those with more activity (5–9 hours/day) [2]. Meanwhile, with the increase of age, inactivity will lead to loss of muscle mass [3], obesity [4], decreased physical fitness ability (PFA) [5], and increased cardiovascular disease (CVD) [6], resulting in reduced capacity of daily activities [7]. Although drug therapy has certain positive effects [8], it also has specific side effects [9]. Therefore, there is a greater need for nonpharmacological treatment of a range of problems for older adults. Furthermore, a lot of evidence from high-quality studies suggests that physical activity improves the health of older adults [10]. Most of the previous studies on traditional Chinese physical activities such as Ba-Duan-Jin, Qigong, and Tai Chi in older adults were about strength, balance, cognition, and hypertension. Meanwhile, all the research studies aimed to improve the PFA and increase the CVD of OF. However, most of their evaluation indicators were reflected in a certain aspect, such as physical fitness, blood pressure, or cardiovascular function. They did not take comprehensive indicators into account.

Tai Chi and TCSB are very similar. Tai Chi has been used as a form of exercise to treat many problems in the elderly, such as strength and balance. Tai Chi softball is a unique Chinese health-promoting exercise invented based on the principle of Tai Chi Quan along with deep breathing and relaxation for promoting internal energy [11]. Tai Chi softball was also voted as one of the most popular health exercises in the category of ball games [12]. Practicing Tai Chi softball is helpful not only for lower extremity physical health. However, it can also develop manipulative skills and hand-eye coordination (eating, dressing, bathing required manipulative skills, grip movement, and strength). Like Tai Chi and TCSB, the combination of some Tai Chi movements with the skills of tennis and badminton is a Tai Chi-style ball game with Chinese tradition. The practice shows that it can improve the symptoms of the patients' exercise performance and improve the quality of patients' life [13]. This was the first time that a traditional Chinese physical activity has been involved. Therefore, it is of great significance to carry out this research.

Aging has always been a genuine concern [14], and as we get older, it brings many problems to our families and society, especially the elderly's own PFA and risk of CVD. However, the primary objective of this study is to check whether the TCSB program could improve physical fitness ability (PFA) and decrease the risk of CVD of OF. Eventually, TCSB may reduce the burden of family and country and improve OF's mental and physical health. The major contributions of this work are as follows:

- This study arranged a 16-week Tai Chi softball (TCSB) training program for older females to study the changes in the physical fitness level and cardiovascular health of older females with and without training
- Biochemical examinations such as total cholesterol (TC), triglycerides (TG), low-density lipoprotein cholesterol (LDL-C), and high-density lipoprotein cholesterol (HDL-C) were performed in a clinical laboratory for all the participants to examine the impact of exercise and training on their health
- The study proved that the Tai Chi softball (TCSB) training program and exercise could significantly reduce the risk of cardiovascular disease and enhance the physical fitness level of older females

The rest of the study is organized as follows: Section 2 describes the methodology of the proposed work.  Section 3 illustrates the results. In Section 4, the results are discussed followed by limitations in Section 5. Finally, Section 6 concludes the study.

## 2. Methods

### 2.1. Study Design

It was a 16-week, nonrandomized, and controlled training intervention trial. The 100 OF participants were recruited from the Xi'an Community-Dwelling Elderly Activity Center. After screening, there were 80 OF who met the criteria. Then, the participants were divided into two groups: the control (C) group and the physical exercise (PE) group according to their wish and physical condition to maximize training effects. Subsequently, the C group and the PE group each had 40 OF. Before the experiment, the physical fitness level and cardiovascular health-related factors were tested. Then, the experimental intervention was carried out. The C group followed their usual lifestyle and routine activities without any intensive physical exercise every day. In contrast, the PE group took 16-week TCSB intervention training. Through 16-week TCSB intervention training, data were collected and analyzed to conclude.

### 2.2. Participants

All the participants were recruited from the Xi'an Community-Dwelling Elderly Activity Center. A total of 100 OF were recruited. The specific criteria that were studied to meet the experiment were included: (1) women who are over 55 years, (2) normal blood pressure, (3) move normally, (4) no major illness, (5) not taking a new drug, and no hospitalizations in the last 3 months. The conditions for exclusion from the experiment were as follows: (1) BMI > 27, (2) high blood pressure disease, (3) lousy eyesight, and (4) dizziness and ringing in the ears during training. Candidates volunteered to participate in the experiment because they had no contraindications to engage in physical activity. Finally, 80 people met the criteria for inclusion. Then, according to the experimental requirements, they were divided into the C group and PE group, respectively. Everyone was informed about the training in advance, and they signed a consent information form.

### 2.3. Intervention

It was a 16-week TCSB intervention experiment. For the first 4 weeks, all PE group participants were required to attend the training for 1 hour per session at 9:30 a.m., four times a week in the Xi'an Community-Dwelling Elderly Activity Center. The training included a 10-minute warm-up, 40-minute TCSB study, and 10-minute cool-down. The TCSB program was divided into two parts. Participants learned first half of the content in the first two weeks and the remaining half in the other two weeks. The process of learning was accompanied by light music. The first four weeks of the intervention aimed to ensure that everyone understood the instructions and could execute the essential TCSB movements. During the subsequent 12 weeks, the time and frequency of training gradually increased. Participants exercised for 1.5 hours every morning at 9:30 a.m. during the 12-week intervention training. The contents consisted of a 20-minute warm-up, 70-minute TCSB training, and a 20-minute cool-down, with 5 sessions a week for a total of 12 weeks. The training place was still the Xi'an Community-Dwelling Elderly Activity Center. The modes involved in TCSB training were from two different TCSB styles (amateur and competitive) of varying degrees of difficulty. The TCSB training was led by one professional. Subjects in this study were required to pause and rest immediately if they experienced any of the following signs or symptoms: shortness of breath, increased discomfort, chest palpitations, dizziness, and/or paleness.

### 2.4. Outcome Measurement

All participants were tested before the trial and after the 16-week TCSB intervention training. The results measurement was based on the physical fitness level test [3, 15–17] and cardiovascular health-related factors [18–23].

#### 2.4.1. Handgrip (HG)

A digital dynamometer with a precision of 0.1 kg was used to measure the HG. Elders stood with the dynamometer held straight down, their shoulders slightly abducted, and their wrist was in a neutral position during the test. Participants were requested and encouraged to use as much force as they could. Each participant repeated the test twice with each dominant side, pausing for at least 30 seconds between each attempt, with the best score being registered (kg).

#### 2.4.2. Sit and Reach (SAR)

The “sit and reach” was tested by using an apparatus. The participants sat on the edge of an apparatus and remained seated on the floor. The upper body was 90 degrees upright, and their legs uncurled. Then, the baffle was touched with one hand to the maximum extent of the front area. The best score was registered after each participant completed the test twice.

#### 2.4.3. Single Leg Stance (SLS)

The timed SLS is an objective measure. Subjects were asked to stand on one leg with their eyes open, arms around their chests, and hands are touching their shoulders during the exercise to see how long subjects could retain SLS stability, and they were timed. Three trials were permitted, and data were collected based on the average time of these trials.

#### 2.4.4. Body Mass Index (BMI) and Waist-to-Hip Ratio (WHR)

The height, bodyweight, and waist-to-hip ratio (WHR) were obtained with an electronic scale and InBody. First, subjects were dressed in light clothing and an empty bladder and stood straight on the electronic scale, and the relevant data were collected. Second, subjects held the InBody handle with both hands (for 30 seconds). Then, the WHR was recorded according to the report. Finally, the BMI was calculated according to their height and weight.

#### 2.4.5. Vital Capacity (VC), Systolic Blood Pressure (SBP), and Diastolic Blood Pressure (DBP)

The vital capacity tester measured vital capacity. The subjects first took a deep breath and then continuously blew towards the instrument nozzle. The maximum value was taken from three measurements. With the participant seated and resting for at least 5 minutes, blood pressure (SDP, DBP) was measured in the nondominant arm.

Biochemical examinations such as total cholesterol (TC), triglycerides (TG), low-density lipoprotein cholesterol (LDL-C), and high-density lipoprotein cholesterol (HDL-C) were performed in a clinical laboratory. Subjects did not drink alcohol and did not do intensity exercise the day before.

### 2.5. Statistical Analyses

The results were analyzed by using the statistical package SPSS 25.0. The data were first tested for normal distribution, and one-way ANOVA was used to compare different groups at the same time. The Kruskal–Wallis H test was used for nonnormal distribution. A paired-sample *t*-test was used to compare before and after the experiment within the same group, and differences were indicated by *p* < 0.05.

## 3. Results

### 3.1. Physical Fitness Level

The physical fitness level was measured before and after the TCSB training intervention.  Figure 1 shows the results of the physical fitness level (mean ± Standard deviation) before and after the TCSB training intervention. It is evident that there was no significant difference in the physical fitness level test of C and PE before the experiment, and PE showed significant differences in their physical fitness after the 16-week TCSB intervention training.

The HG, SAH, and SLS in PE, the average physical fitness level and standard deviations, were 27.5 ± 5.1 (kg), 11.9 ± 5.71 (cm), 11.1 ± 5.82 (s) respectively. After the 16-week intervention training, HG, SAH, and SLS were 31.25 ± 5.15 (kg), 13.78 ± 6.28 (cm), and 14.72 ± 7.33(s). It was concluded that the HG, SAH, and SLS increased by 13.6%, 24%, and 32.6%, respectively, which is a significant difference (^*∗*^*p* < 0.05).

### 3.2. Cardiovascular Health

In the cardiovascular health test, nine indicators were included. As shown in Figure 2, there was no significant difference in the cardiovascular health of the C and PE groups before the experiment. However, after the 16-week TCSB intervention training, the PE group showed significant differences.

The BMI and WHR in the PE group were 25.82 ± 2.1 (kg/m^2^) and 0.94 ± 0.08 respectively. After the 16-week TSCB intervention training, BMI and WHR were reduced to 25.32 ± 2.1 (kg/m^2^) and 0.9179 ± 0.07. The reduction in BMI and WHR clearly showed a significant difference (^*∗*^*p* < 0.05) in the cardiovascular health of the two groups. Similarly, VC, SBP, and DBP in the PE group before the intervention were 1766 ± 301 (ml), 136 ± 16.9 (mmHg), and 83 ± 10.1 (mmHg), respectively. After intervention training, VC, SBP, and DBP recorded was 1974 ± 447 (ml), 132 ± 15 (mmHg), and 78.79 ± 8.39 (mmHg), respectively. The SBP and DBP showed a significant difference (^*∗*^*p* < 0.05). However, VC showed a more significant difference (^*∗∗*^*p* < 0.01) in cardiovascular health. In the case, TC, TG, HDL-C, and HDL-C in the PE group before the intervention were 4.33 ± 0.96 (mmol/L), 2.22 ± 1.74(mmol/L), 1.19 ± 0.22 (mmol/L), and 2.76 ± 0.68 (mmol/L), respectively, but after training, the TC, TG, HDL-C, and HDL-C reported were 4.06 ± 0.92 (mmol/L), 1.3 ± 0.64 (mmol/L), 1.29 ± 0.21 (mmol/L), and 2.51 ± 0.59 (mmol/L). The TC, TG, and HDL-C showed a significant difference (^*∗*^*p* < 0.05). However, HDL-C showed a more prominent difference (^*∗∗*^*p* < 0.01) in their cardiovascular health.

## 4. Discussion

This research proved that the strength, flexibility, balance, vital capacity, blood pressure, and lipids of OF were improved in the 16-week TCSB intervention training. In this experiment, great emphasis was put on two major parts. The first part was the effect of the 16-week TCSB intervention training on HG, SAH, and SLS of OF. The second part was the effect of the 16-week TCSB intervention training on VC, HR, SBP, DBP, TC, TG, HDL-C, and LDL-C of the older females. Conclusively, the 16-week TCSB intervention training increased the PFA and decreased the CVD risk of OF.

In the physical fitness level test, HG has revealed an improvement of 13.6% after the 16-week TCSB intervention training compared with that before the intervention. Meanwhile, the result was similar to those reported by Sousa et al. [24] and Halder et al. [25]. The main reason was that the regular use of the Tai Chi handle can improve the regulation of the nervous system. It increases the ability of the central nervous system to recruit peripheral motor unit activities. It improves the degree of synchronization of motor unit activities and the coordination of the activities of different muscle groups. The same was confirmed that the postintervention SAH had revealed an improvement of 24% compared with that before the intervention. Our results also match with the study given in [15]. The wide range of motion of the arms, shoulders, hips, and knees in multiple directions was the main reason for the increased flexibility during the 16-week TCSB intervention training. In the previous research findings, exercise can improve balance [18]. In our study, the postintervention SLS has revealed an improvement of 32% compared with that before the 16-week TCSB intervention training. In TCSB training, there were often many movements, such as turning around and standing on one foot. The long-term training will stimulate the sensory cells of the vestibular organs to produce nerve impulses, which are transmitted to the central nerve via the vestibular nerve. It causes the body to feel its position in space and maintain body balance.

In summary, the 16-week TCSB training can improve older females' strength, flexibility, and balance. Furthermore, physical training can strengthen older females' physical exercise ability. Previous studies have shown that exercise can reduce weight and waist circumference [26]. In our study, however, the BMI and WHR were 25.32 ± 2.1 and 0.9179 ± 0.07, respectively, in the 16-week TCSB intervention training, and they had significant differences. Our results were similar to those of others researchers [27], but other studies showed that older adults with a high BMI might be presumed to have CVD risk. Similarly, WHR was one of the factors leading to CVD [28]. There were two significant reasons for these results. On the one hand, in the 16-week TCSB intervention training, OF have more rotation movements. On the other hand, in the 16-week TCSB intervention training, OF have systematic long-term endurance training. Therefore, the risk of CVD can be reduced in OF through TCSB training.

It was a very common fact that exercise can decrease high blood pressure [29]. Our results in this research were the same as the previous study. Both SBP and DBP decreased and showed a significant difference. Notably, blood pressure is an important indicator of CVD, and high blood pressure increases CVD risk [30]. Therefore, the 16-week TCSB intervention training can help prevent CVD and reduce the risk of CVD. Long-term TCSB training keeps the elasticity of the walls of small arteries from weakening with the passage of time and can maintain good elasticity. With the decrease of sympathetic tension at rest, the impulse issuance of sympathetic constrictor nerves to small arterial vessels is correspondingly weakened, so the peripheral resistance is smaller, allowing blood pressure to fall.

Furthermore, exercise has a protective effect against many of the recognized risk factors for CVD, including hypertension, dyslipidemia, and type 2 diabetes [31]. Among all CVD, TC, TG, HDL-C, and LDL-C are the most important. Furthermore, the change of TC, TG, HDL-C, and LDL-C largely determined the probability of CVD. Our findings on TC, TG, HDL-C, and LDL-C display a significant improvement in the 16-week TCSB intervention training. Meanwhile, physical training, for example, reduces TC, TG, and LDL-C and raises HDL-C [18]. Our results agree with those reports. In conclusion, physical activity can reduce CVD risk, and the 16-week TCSB intervention training can improve cardiovascular function.

## 5. Limitations

The experimental subjects were all older females, while some older males should have been recruited. The intensity of the experiment was not controlled, leading to discomfort in some of the older adults, such as dizziness and vomiting. The variables tested were selected only for significant differences, and no corresponding explanations were given for reaction time, core strength, or heart rate.

## 6. Conclusion

The proposed study explored changes in the physical fitness level and cardiovascular health-related factors among older females after the 16-week Tai Chi softball (TCSB) training program. One hundred healthy older females were assessed at the baseline before TCSB training, and they conducted intervention experiments. Our results showed that TSCB training could improve older females' strength (HG), flexibility (SAH), and balance (SLS). Furthermore, it can improve their PFA. Meanwhile, it also enhanced their cardiovascular function and reduced the risk of CVD. Therefore, TSCB deserves to be applied to more communities to serve the elderly. It can be an effective means to reduce CVD and enhance cardiovascular function.

## Figures and Tables

**Figure 1:** Comparison diagram of physical fitness level data results in (a) HG, (b) SAR, and (c) SLS.

**Figure 2:** Comparison diagram of cardiovascular health-related factors results.

## Data Availability

The data used to support the findings of this study are included within the article.
